# Does Income Inequality Harm Green Growth? The BRICS Experience

This article has been retracted.

**DOI:** 10.1155/2022/7046208

**Published:** 2022-10-12

**Authors:** Wanling Chen, Shaoming Chen, Yuping Tang

**Affiliations:** ^1^Research Center for International Trade and Economics, Guangdong University of Foreign Studies, Guangzhou 510006, China; ^2^School of Economics, Guangzhou City University of Technology, Guangzhou 510800, China; ^3^International Business School, Guangzhou City University of Technology, Guangzhou 510800, China

## Abstract

Green growth plays a vital role in ensuring sustainable development. Managing economic growth without disrupting the environment is considered the need of the present time. Therefore, the empirics have turned their attention toward finding the determinants of green growth. Hence, we aim to investigate the impact of income inequality on green growth in BRICS economies from 1993 to 2020. Findings of the panel autoregressive distributed lag (ARDL) model confirm that the long-run estimate attached to GINI is negatively significant, implying that higher inequality in the BRICS economies lowers the rate of green growth. The country-wise results highlighted the negative impact of GINI on green growth in India and China only and insignificant in other countries. In the short run, the estimates are inconclusive and mixed, be it group-wise or individual estimates. Our findings imply that the target of lower inequality and environmental sustainability can be achieved simultaneously.

## 1. Introduction

Sustainable development of ecological, social, and economic life for forthcoming generations necessitates the right decision-making from today. In this perspective, endorsing sustainable growth has become a fundamental objective for all economies. In order to attain sustainable growth, 129 member states of the United Nations (UN) designated “2030 sustainable development strategy” in 2015 [1]. This strategy aims to achieve several objectives such as the establishment of strong institutions, enhancement of environmental quality, and reduction in inequalities and poverty. Furthermore, it aims to solve fundamental environmental, social, and economic issues [2]. It is frequently revealed that deteriorating environmental quality and income inequality are two imperative complications to sustainable growth [3]. The United Nations also emphasizes that inequalities and environmental degradation are the two most important matters of the current time, and solution for these issues on a priority basis is necessary for sustainable green growth [4].

Sachs [5] highlighted that the global economy has attained substantial achievement in endorsing economic development but has not obtained the same achievement in terms of environment and welfare distribution. Consequently, it can be claimed that income inequality is a fundamental hindrance to the development of harmonious societies. Since 1980s, the speedy worsening of income distribution has become the main socioeconomic issue [6]. The speedy worsening of income distribution led to an increased investigation of the dynamics of income inequality in developing and developed economies. Most specifically in the OECD economies and in US, income inequality has deteriorated speedily since the last few years [7]. This speedy deterioration of income inequality has influenced the wealth distribution dynamics. For instance, the share of the upper 0.1 percent cluster in total wealth enlarged from 7 percent in 1987 to 22 percent in 2012 in the USA. Additionally, deterioration in income distribution has also been observed in developing economies as well during the neoliberal era. For example, Banerjee and Piketty [8] conveyed that the share of the upper 1 percent cluster in total wealth has enlarged during the period of economic liberalization in India. In the recent era, income inequality has significantly increased in China [9].

Another reason behind unsustainable development is a deterioration of environmental quality [10]. The global rise in consumption and production has increased energy consumption and natural resource consumption. The increased consumption of fossil fuels, the more globalized economic relations, and the increased world population have raised environmental pressure and instigated fundamental changes in the ecosystem. An increase in consumption of fossil fuels such as natural gas, coal, and crude oil accounts for approximately 75 percent of energy use, which mitigates the efficiency of energy and causes major environmental problems [11]. An increase in greenhouse gas emissions in the form of CO2 from the consumption of fossil fuels is the main determinant of environmental deterioration, such as climatic change and global warming. Global CO2 emissions are rising rapidly in recent years, and it is predicted that the climatic pressure will raise more if CO2 emissions could not be controlled [12]. For this reason, the needs for green growth, energy efficiency, and CO2 emission reduction have become tactical determinants for attaining sustainable development objectives.

Due to the upsurge in environmental disasters, green growth has become a strategic choice for the attainment of sustainable development [13]. The green growth concept has motivated widespread concerns and is considered an effective source of saving resources, raising growth, and mitigating environmental issues [14]. Research organizations have developed proper definitions for green growth and considered it a strategic idea [15]. Loiseau et al. [16] identified the characteristics and dimensions of green growth and examined the association between economic sustainability and green growth. There are several other studies discussing the concept of green growth. Musango et al. [14] claimed that conversion towards green growth can save natural resources and reduce CO2 emissions. Reilly [17] revealed that job creation, protection of the environment, and economic growth are three core purposes of green growth. Additionally, Bagheri et al. [18] investigated green growth potential for Canada, Ma et al. [19] explored green growth efficiency for China, and Yang et al. [20] investigated green growth differences for various resource-intensive regions of China.

In recent years, increasing concern over income inequality and environmental degradation has raised a new aspect to the literature of environmental issues by linking socioeconomic inequalities with environmental problems [21, 22]. Under this perspective, it has become an imperative research query whether income inequalities influence environmental degradation. Within this context, researchers aim to search the impact of income inequalities dynamics on indicators of the environment such as air pollution, water pollution, ecological deficit, and CO2 emissions and added new dimensions to the literature [23]. Although several studies have been done on this area, but no empirical and theoretical consensus has been gained yet. Baek and Gweisah [24] and Uzar and Eyuboglu [22] reveal that environmental issues are social issues stemming from power and income inequalities; however, few researchers such as Grunewald et al. [25] describe that income inequality has no impact on environmental quality.

It can be observed that there exists vast literature elaborating on the connection between income distribution and environmental quality. However, the effect of income distribution on green growth which imperative catalyst in improving environmental sustainability and reducing carbon dioxide emissions has been neglected in the literature. In fact, in the modern era, initiatives to classify the main factors of green growth have increased speedily. In literature, it is observed that political, environmental, and economic variables such as education [26], technology [27], green finance [28], trade openness [29], R&D [30], environmental regulations [31], and fiscal spending [32] are considered as primary determinants of green growth. However, current literature neglects a fundamental determinant of green growth such as income inequality which causes the socioecological part of the energy and environmental studies. From this perspective, the present study aims to identify the impact of income inequalities on green growth in the case of BRICS economies for time period 1993-2020. This study answers the question “is the income inequality harms green growth?” As far as the authors' knowledge is concerned, this is the first study to investigate the influence of income inequality on green growth in the context of BRICS. This study employs the ARDL-PMG approach to capture long- and short-run nexus between income inequality and green growth. The results of this study will benefit in designing environmental sustainability policies.

## 2. Model and Methods

Theoretically, income inequality may have a negative or positive effect on CO2 emissions, which may have an impact on the sustainable economic development of the economy. The income inequality estimate on environmental quality mainly depends on the nexus between demand-income. In the case of the linear relationship between demand-income, any transfer of money from poor to rich will not have any impact on the environmental quality [33, 34]. On the other side, if the demand-income relationship follows a convex path, then a single penny transfer from poor to rich will significantly impact the environmental quality [35]. If income inequality strongly impacts CO2 emissions, we believe that it also affects production-based CO2 emissions, i.e., green growth [36, 37]. Hence, we have developed the following model.

(1) $$\begin{array}{c} {\text{GG}}_{\text{it}}=\varphi_{0}+\varphi_{1}{\text{GINI}}_{\text{it}}+\varphi_{2}{\text{EI}}_{\text{it}}+\varphi_{3}{\text{Education}}_{\text{it}}+\varphi_{4}{\text{GS}}_{\text{it}}+\varphi_{5}{\text{FD}}_{\text{it}}+\varepsilon_{\text{it}}, \end{array}$$

where green growth (GG) is a dependent variable, which is determined by income inequality (GINI), environmental innovations (EI), average years of schooling (Education), government spending (GS), financial development (FD), and error term (*ε*_it_). Equation (1) presents only long-run estimates. The short-run effects are also equally important to explore. To this end, we follow Pesaran et al. [38] error correction format:

(2) $$\begin{array}{c} {\Delta \text{GG}}_{\text{it}}=\varphi_{0}+\overset{p}{\underset{i=1}{\sum }}\pi_{1\text{k}}{\Delta \text{GG}}_{\text{it}-\text{i}}+\overset{p}{\underset{i=0}{\sum }}\pi_{2k}{\Delta \text{GINI}}_{\text{it}-i}+\overset{p}{\underset{i=0}{\sum }}\pi_{3k}{\Delta \text{EI}}_{\text{it}-i}+\overset{p}{\underset{i=0}{\sum }}\pi_{4k}{\text{Education}}_{\text{it}-i}+\overset{p}{\underset{i=0}{\sum }}\pi_{5k}{\text{GS}}_{\text{it}-i}+\overset{p}{\underset{i=0}{\sum }}\pi_{6k}{\text{FD}}_{\text{it}-i}+\varphi_{1}{\text{GG}}_{\text{it}-1}+\varphi_{2}{\text{GINI}}_{\text{it}-1}+\varphi_{3}{\text{EI}}_{\text{it}-1}+\varphi_{4}{\text{Education}}_{\text{it}-1}+\varphi_{5}{\text{GS}}_{\text{it}-1}+\varphi_{6}{\text{FD}}_{\text{it}-1}+\lambda .{\text{ECM}}_{\text{it}-1}+\varepsilon_{\text{it}}. \end{array}$$

Equation (2) is called the ARDL-PMG framework and was proposed by Pesaran et al. [38]. The panel cointegration test is used to examine long-run relationships among economic variables. Pesaran et al. [38] proposed the *F*-test and ECM test for cointegration. The panel ARDL has several benefits. This method is more feasible at different orders of integration, such as I(0), I(1), or a mix of both types of variables (Bahmani-Oskooee et al., 2020). So for that, our study has used LLC, IPS, and ADF unit root tests. Panel ARDL also accommodates small samples. The panel ARDL simultaneously estimates both short- and long-run effects. The long-run effects are derived from *φ*_2_ − *φ*_6_ by normalizing on  *φ*_1_, while the short-run effects in the above-mentioned Equation (2) are identified by first-differenced signs. The ARDL panel technique takes into account the endogeneity and serial correlation issues.

The study explores the impact of income inequality on green growth in the case of BRICS economies. The impact of income inequality on green growth is determined by controlling the effect of education, environmental innovation, government spending, and financial development. The details regarding variables' definitions, symbols, and data sources are given in Table 1. Green growth (GG) is measured through environmentally adjusted multifactor productivity. Income inequality is determined through the GINI index. The control variables are selected based on previous green growth literature [27, 39]. Secondary school enrolment is taken to measure education. Environmental innovation is measured via the development of environment-related technologies as percent of all technologies. Government spending is taken as general government final consumption expenditures as percent of GDP. Financial development is taken as domestic credit to private sector as percent of GDP. The data for the empirical analysis is taken from OECD and the World Bank. The mean (S.D) of GG, GINI, Education, EI, GS, and FD are 5.096% (3.313%), 1.652 (0.100), 1.909% (0.114%), 9.174% (2.561%), 16.25% (3.185%), and 1.760% (0.329%), respectively (Table 2).

## 3. Results and Discussion

To make and perform an empirical task, our study employed panel and time-series ARDL techniques for panel-wise and economy-wise analysis. As a first step, it is essential to check the stationarity properties of variables. In Table 3, according to LLC unit root test, it is found that GINI and GS are integrated at I(0) while GG, education, EI, and FD are integrated at I(1). However, IPS and ADF-Fisher tests produce similar results. It is found that EI and GS are stationary at I(0) and GG; GINI, Education, and FD are stationary at I(1).  Table 4 displays the economy-specific and panel-specific results of long-term and short-run parameters of green growth models.

In the panel-specific model, the findings infer that an increase in GINI tends to reduce green growth, depicting that increase in income inequality results in reducing green growth in the panel of BRICS economies. It reports that a 1% upsurge in GINI causes 3.126% reduction in green growth in the long-term. The empirical analysis confirmed that higher income inequality leads to low green growth. Some other findings, such as Hallegatte et al. [40], Fay [41], and Kim et al. [42], also suggest that lower-income inequality means low emissions of CO2 during production activities. However, some other empirical suggests otherwise. For instance, Liu et al. [43] and Huang and Duan (2020) confirm that higher income inequality leads to low CO2 emissions during production and consumption activities. Empirical evidence suggests that the environmental impacts of income inequality are more prominent in developing economies than the developed economies. This is because the higher income inequality in developing economies is a barrier to the ubiquity of innovation, which hinders the development of green technological innovation.

Furthermore, the wide gap between the poor and the rich in developing economies induces policymakers to divert the flow of resources from research and development activities to the social security benefits programs. As a result, the firms have to rely on obsolete methods of production that take the economy further away from the target of green growth [44]. Moreover, the higher gap between rich and poor people also leads to a low literacy rate in developing economies, which means less awareness about the harmful impact of environmental degradation [45] and green growth. In developed economies, the income distribution is more equitable, which is suitable for developing environment-related technologies and green products. Besides, it also helps to introduce more relevant environment-related regulations [44]. The impact of the GINI coefficient is not significant on the CO2 emissions in developed economies; however, in the countries where per capita income is too high, evidence suggests a negative correlation between the GINI coefficient and environmental quality. Conversely, McGee and Greiner [46] demonstrated that income inequality might help reduce CO2 emissions during industrial and manufacturing activities in smaller developed economies.

Education reports an increasing impact on green growth in the long-term, confirming that an increase in education escalates green growth in BRICS economies. A 1% increase in the level of education causes 2.678% upsurge in green growth. Environmental innovation raises green growth in the long-term, displaying that increase in eco-innovation is useful to attain green growth in BRICS economies. It reveals that 1% rise in environmental innovation increases green growth by 0.187% in the long-term. In the long-term, government spending does not report a significant association with green growth in the BRICS economies. Conversely, financial development increases green growth, confirming that access of financial resources significantly contributes in increasing green growth in BRICS economies. It reports that 1% expansion in financial development causes 1.629% upsurge in green growth in the long-term. The short-term results show that GINI does not report a significant association with green growth. However, education, environmental innovation, and financial development report significant increases in green growth in the panel of BRICS economies.

In the economy-specific models, the long-run findings reveal that GINI reduces green growth in two economies of BRICS, depicting that increase in income inequality leads to a reduction in green growth in the long-term. A 1% increase in GINI causes a decline in green growth by 0.828% in India and 1.974% in the long-term. However, education enhances green growth in two of BRICS economies, describing that increase in level of education tends to improve the green growth in BRICS countries. A 1% improvement in education causes increase in green growth by 1.498% in India and 1.308% in China. Environmental innovation also results in the enhancement of green growth in three of BRICS countries. It confirms that eco-innovation acts as a vital measure that improves green growth in BRICS economies. It shows that a 1% increase in environmental innovation tends to enhance green growth by 1.492% in Russia, 1.140% in China, and 0.358% in South Africa. Government spending shows a positive enhancement in green growth in three BRICS economies in the long-term, confirming the significant role of government spending in enhancing green growth. It displays that a 1% rise in government spending ensures an upsurge in green growth by 1.485% in Russia, 1.482% in India, and 0.684% in China. In the end, financial development enhances green growth in two economies only displaying that 1% upsurge in financial development increases green growth by 1.424% in Brazil and 1.372% in India in the long-term. The short-run findings describe that GINI reduces green growth in India and China, confirming the negative association between income inequality and green growth. Education is positively attached with green growth in India only in the short-term. Environmental innovation increases green growth in China only. Government spending tends to reduce green growth in India only in the short-term. Financial development enhances green growth in Brazil, India, and China in the short-term.

In the end, some diagnostic test results are given, which are required to confirm the validity of ARDL results. The *F*-test and ECM test confirm the cointegration association among variables in the long-term. The stability condition is fulfilled through the both CUSUM tests. Finally, in Table 5, the results of the causality test for the BRICS nations panel and economy-wise show that unidirectional causality exists between GINI and GG in BIRCS, India, and China, while causality does not exist from GINI to GG in Brazil, Russia, and South Africa.

## 4. Conclusion and Implications

Environmentalists have observed that the increase in worldwide production and consumption activities has contributed massively to climate change due to emissions of greenhouse gasses. Over the past few decades, the world has witnessed unprecedented changes in the climate, including high temperatures, melting glaciers, storms, floods, and droughts. Such climate changes have rung the alarm bells for this generation and the upcoming generations. Therefore, the issue of climate change and global warming has become the buzzword in the 21^st^ century and the most debated topic at international conferences. In this regard, the world community has signed treaties. The main crux of such treaties is preserving the environment for future generations by controlling CO2 emissions. As a result, the concept of green growth has emerged, which decouples economic growth from CO2 emissions. Recently, the empirics have turned their attention towards finding the determinants of green growth. However, the impact of income inequality on green growth is yet to be explored. Hence, we aim to investigate the impact of income inequality on green growth in BRICS economies.

To investigate empirically, we have first applied unit root tests, including LLC, IPS, and ADF-Fisher, which imply that series are a mixture of I(0) and I(1). Findings of the ARDL-PMG model confirm that the long-run estimate attached to GINI is negatively significant and implies that higher inequality in the BRICS economies lowers the rate of green growth. The country-wise results highlighted the negative impact of GINI on green growth in India and China only and insignificant in other countries. Among the control variables, the estimates of Education, EI, and FD are positively significant, suggesting that education, environmental innovations, and financial development promote green growth in the long run. In the short run, the estimates are inconclusive and mixed, whether group-wise or individual.

In order to reduce environmental pollution, we can propose some policy recommendations. Our findings suggest that high-income inequality in BRICS economies is detrimental to green growth. Therefore, we can confer that lower-income inequality and environmental sustainability targets can go side by side in BRICS economies. Therefore, policymakers should try to promote policies that can bring more income equality by taking various steps, such as social security benefits to the poor, tax policy reforms, and creating employment opportunities for a deprived faction of the society. All these policies not only help to reduce income inequality but also help in environmental sustainability as well green growth.

Since the analysis has contributed to the literature in many ways, it still has shortcomings. First, the analysis only covers BRICS economies, and the inference drawn from the study is only valid for developing economies. However, the issue of income inequality is more severe in less developing economies; therefore, the empirics should investigate the analysis for underdeveloped economies in the future. Moreover, the empirical research does not account for the cross-section dependence, and future studies should consider the techniques that can handle the issue of cross-sectional dependence.

## Figures and Tables

**Table 1:** Definitions and data sources.

Variable	Symbol	Definitions	Sources
Green growth	GG	Environmentally adjusted multifactor productivity	OECD
GINI	GINI	Gini index	World bank
Educational attainment	Education	School enrolment, secondary (% gross)	World bank
Environmental innovation	EI	Development of environment-related technologies, % all technologies	OECD
Government spending	GS	Government final consumption expenditure (% of GDP)	World bank
Financial development	FD	Domestic credit to private sector (% of GDP)	World bank

**Table 2:** Descriptive statistics.

	Observations	Mean	Median	Max	Min	S.D.	Skewness	Kurtosis
GG	140	5.096	4.930	13.13	-6.233	3.313	-0.513	3.930
GINI	140	1.652	1.612	1.812	1.501	0.100	0.289	1.491
Education	140	1.909	1.958	2.041	1.634	0.114	-1.047	2.905
EI	140	9.174	9.271	16.80	3.730	2.561	0.230	2.447
GS	140	16.25	16.98	21.07	9.802	3.185	-0.692	2.239
FD	140	1.760	1.743	2.261	0.456	0.329	-0.951	4.268

**Table 3:** Unit root tests.

	LLC		IPS		ADF-fisher	
	I(0)	I(1)	I(0)	I(1)	I(0)	I(1)
GG	-0.231	-4.056^∗∗∗^	-0.012	-4.078^∗∗∗^	-0.012	-4.187^∗∗∗^
GINI	-2.198^∗∗^		-0.178	-2.055^∗∗^	-0.254	-2.879^∗∗∗^
Education	0.102	-3.587^∗∗∗^	1.821	-3.875^∗∗∗^	1.954	-3.897^∗∗∗^
EI	-1.023	-6.023^∗∗∗^	-1.654^∗^		-1.534^∗^	
GS	-2.356^∗∗∗^		-3.452^∗∗∗^		-3.321^∗∗∗^	
FD	-0.345	-3.875^∗∗∗^	0.402	-5.345^∗∗∗^	0.465	-5.012^∗∗∗^

Note: ^∗∗∗^*p* < 0.01; ^∗∗^*p* < 0.05; ^∗^*p* < 0.1. Source: Author estimations.

**Table 4:** Green growth estimates.

Variable	BRICS		Brazil		Russia		India		China		South Africa	
	Coefficient	*t*-stat	Coefficient	*t*-stat	Coefficient	*t*-stat	Coefficient	*t*-stat	Coefficient	*t*-stat	Coefficient	*t*-stat
Long-run												
GINI	-3.126^∗^	-1.726	1.813	0.963	1.042	1.093	-0.828^∗∗^	-2.511	-1.974^∗∗^	-2.428	-0.114	-1.088
Education	2.678^∗∗∗^	4.360	2.899	0.799	1.835	0.658	1.498^∗∗^	2.285	1.308^∗∗^	2.281	2.915	1.126
EI	0.187^∗∗^	2.082	0.136	0.284	1.492^∗∗∗^	4.049	0.483	1.277	1.140^∗^	1.701	0.358^∗^	1.695
GS	0.103	0.579	0.477	0.651	1.485^∗∗∗^	5.005	1.482^∗∗∗^	3.170	0.684^∗^	1.878	-0.590	-0.930
FD	1.629^∗^	1.705	1.424^∗∗^	2.335	1.550	0.919	1.372^∗^	1.910	4.875	1.379	1.809	0.587
Short-run												
D (GINI)	-2.050	-0.971	0.608	0.988	1.827	1.136	-0.353^∗^	-1.914	0.935^∗∗∗^	2.783	-1.455	-0.125
D (GINI (-1))	1.137	1.064					-0.007^∗∗^	-2.267			-1.043	-1.098
D (GINI (-2))	0.070	1.189					-0.744	-1.380			-1.801	-1.570
D (Education)	-1.333^∗∗∗^	-4.808	-1.327	-0.679	1.467	0.677	1.082^∗∗∗^	3.338	0.598	1.589	0.553	1.111
D (Education (-1))	-0.513	-1.161	-1.088	-0.508					0.147	1.149	0.437	1.250
D (Education (-2))	-0.549^∗∗^	-2.151	0.245^∗∗^	2.259					0.091^∗∗∗^	3.130		
D (EI)	0.304^∗^	1.769	0.568	1.120	0.261	0.797	-0.289	-0.830	0.210^∗∗∗^	2.709	0.090	0.713
D (EI (-1))	0.152	0.781	0.143	0.256	0.659^∗∗^	2.350	0.217	0.942				
D (EI (-2))	0.127	0.550	0.599	1.358	0.994^∗∗∗^	3.792	0.618^∗∗^	2.301				
D (GS)	-0.221	-0.565	-0.609	-0.668	-0.546	-1.464	-1.998^∗∗^	-2.106	-0.953	-1.253	0.262	0.447
D (GS (-1))	-0.116	-0.421			-0.359^∗∗∗^	-3.053	0.316	0.255	0.912	1.075	-0.555	-0.905
D (GS (-2))	-0.125	-0.690					-2.257^∗∗∗^	-2.644	-0.985	-1.487	0.918	1.654
D (FD)	1.235^∗^	1.808	1.582^∗∗^	2.367	1.089	0.871	1.623^∗∗∗^	3.159	2.405^∗∗^	2.184	1.237	0.608
D (FD (-1))	1.158^∗∗∗^	5.774					0.305^∗∗∗^	2.589	1.842	0.546	2.016^∗∗^	2.126
D (FD (-2))	0.080	0.012					0.597	0.948	1.726^∗∗^	2.475	2.796^∗∗^	2.332
C	3.210^∗∗∗^	3.447	6.390	1.111	3.324^∗∗^	2.397	5.998^∗∗^	2.329	2.463^∗∗∗^	3.112	3.247^∗^	1.949
Diagnostics												
*F*-test	6.554^∗∗∗^		6.542^∗∗∗^		10.02^∗∗∗^		6.645^∗∗∗^		7.023^∗∗∗^		2.754	
ECM (-1)	-0.651^∗∗∗^	-3.658	-0.568^∗∗^	-2.126	-0.546^∗∗^	-2.141	-0.314^∗∗∗^	-8.624	-0.498^∗∗∗^	-8.773	-0.523^∗∗∗^	-5.010
LM			1.023		0.655		2.002		0.987		1.875	
Reset			0.987		0.775		1.012		1.987		0.879	
CUSUM			S		S		S		S		S	
CUSUM-sq			S		S		S		S		S	

Note: ^∗∗∗^*p* < 0.01; ^∗∗^*p* < 0.05; ^∗^*p* < 0.1. Source: Author estimations.

**Table 5:** Results of causality test.

Null hypothesis:	BRICS		Brazil		Russia		India		China		South Africa	
	*F*-stat	Prob.	*F*-stat	Prob.	*F*-stat	Prob.	*F*-stat	Prob.	*F*-stat	Prob.	*F*-stat	Prob.
GINI → GG	4.480	0.013	2.277	0.127	0.984	0.391	2.955	0.074	4.702	0.021	2.174	0.139
GG → GINI	0.090	0.914	0.042	0.959	0.153	0.859	0.945	0.405	0.631	0.542	0.226	0.799
EDUCATION → GG	2.961	0.074	1.809	0.188	1.097	0.352	3.114	0.065	2.583	0.099	2.022	0.157
GG → EDUCATION	2.181	0.117	0.503	0.612	0.531	0.596	2.734	0.088	2.757	0.087	0.387	0.684
EI → GG	2.879	0.060	2.505	0.106	8.301	0.002	0.518	0.603	0.701	0.507	0.114	0.893
GG → EI	0.477	0.622	0.246	0.784	0.305	0.740	3.262	0.058	2.315	0.123	0.615	0.550
GS → GG	8.451	0.000	0.042	0.959	4.277	0.028	1.607	0.224	0.868	0.434	3.793	0.039
GG → GS	1.492	0.229	0.659	0.528	0.852	0.441	1.575	0.231	2.944	0.075	1.785	0.192
FD → GG	1.141	0.323	0.739	0.490	0.462	0.636	2.483	0.108	0.387	0.684	4.716	0.020
GG → FD	0.465	0.629	1.201	0.321	0.056	0.945	3.854	0.038	10.74	0.001	0.094	0.911
Education → GINI	3.327	0.039	1.003	0.384	3.129	0.065	0.499	0.614	1.081	0.358	0.921	0.414
GINI → Education	1.652	0.196	0.035	0.965	6.153	0.008	5.491	0.012	1.333	0.285	1.262	0.304
EI → GINI	0.479	0.620	1.298	0.294	0.662	0.526	2.265	0.129	0.933	0.409	0.523	0.600
GINI → EI	2.896	0.059	3.522	0.048	1.410	0.266	10.97	0.001	0.873	0.432	3.210	0.061
GS → GINI	2.417	0.093	0.304	0.741	0.302	0.742	0.376	0.691	0.583	0.567	2.077	0.150
GINI → GS	1.684	0.190	0.242	0.788	0.913	0.417	1.378	0.274	0.084	0.919	2.380	0.117
FD → GINI	2.124	0.124	0.646	0.534	1.434	0.261	2.184	0.138	1.117	0.346	2.630	0.096
GINI → FD	1.407	0.249	7.335	0.004	2.839	0.081	4.336	0.027	0.236	0.792	4.268	0.028
EI → Education	0.045	0.956	0.408	0.670	0.703	0.506	0.243	0.786	0.187	0.831	0.501	0.613
Education → EI	2.621	0.077	0.437	0.652	5.924	0.009	7.809	0.003	0.190	0.829	0.367	0.697
GS → Education	0.020	0.981	0.129	0.880	0.532	0.595	1.941	0.169	0.610	0.553	0.590	0.563
Education → GS	2.921	0.058	0.314	0.734	0.165	0.849	1.049	0.368	2.862	0.080	5.808	0.010
FD → Education	3.532	0.032	0.306	0.740	0.805	0.460	10.13	0.001	2.325	0.122	0.465	0.635
Education → FD	0.109	0.897	0.533	0.595	0.062	0.940	2.257	0.129	3.506	0.049	1.007	0.382
GS → EI	0.669	0.514	1.184	0.326	0.539	0.591	1.954	0.167	2.017	0.158	1.020	0.378
EI → GS	1.327	0.269	0.553	0.584	1.123	0.344	1.061	0.364	0.508	0.609	1.529	0.240
FD → EI	0.589	0.556	3.721	0.041	0.036	0.965	13.86	0.000	0.189	0.829	0.821	0.454
EI → FD	0.507	0.603	3.230	0.060	1.247	0.308	5.233	0.014	0.742	0.488	3.420	0.052
FD → GS	1.241	0.293	9.499	0.001	0.447	0.645	1.900	0.175	2.585	0.099	9.282	0.001
GS → FD	0.311	0.733	1.658	0.215	0.105	0.901	0.592	0.562	0.063	0.939	0.137	0.872

Source: Author estimations.

## Data Availability

The data used to support the findings of this study are available from the corresponding author upon request.
